# An Effective Approach of Vehicle Detection Using Deep Learning

**DOI:** 10.1155/2022/2019257

**Published:** 2022-07-30

**Authors:** Yidan Chen, Zhenjin Li

**Affiliations:** ^1^School of Physics and Electronic Science, Changsha University of Science & Technology, Changsha,410114, China; ^2^School of Foreign Language, Hunan University of Finance and Economics, Changsha 410205, China

## Abstract

With the rise of unmanned driving and intelligent transportation research, great progress has been made in vehicle detection technology. The purpose of this paper is employing the method of deep learning to study the vehicle detection algorithm, in which primary-stage target detection algorithms, namely, YOLOv3 algorithm and SSD algorithm, are adopted. Therefore, the method first processes the image data in the open-source road vehicle dataset for training. Then, the vehicle detection model is trained by using YOLOv3 and SSD algorithms to show the detection effect, respectively. The result is by comparing the detection effects of the two models on vehicles. The researchers accomplished the result analysis and summarized the characteristics of various models obtained by training, to apply to target tracking, semantic segmentation, and unmanned driving.

## 1. Introduction

In recent years, artificial intelligence technology with deep learning as its core has also made considerable progress, among which deep learning is employed as the core technology in computer vision field. Target detection technology, as one of the core technologies in the field of computer vision, provides basic technical support for many aspects, such as target tracking, semantic segmentation, and unmanned driving.

Unmanned driving system is constituted by three parts: perception, planning, and control. Perception refers to perceiving the surrounding environment. Specifically, it can be classified into perception of things and perception of people. Perception of things further incorporates perception of vehicles and perception of obstacles. In the unmanned driving system, the computer vision technologies are used to perceive the environment mainly by detecting the surrounding environment through the target detection technology. Of course, other sensors are also applied to perceive the environment. The advent of automatic parking system embodies the vehicle's perception of the surrounding environment. Many scientific technologies, including machine vision, are used to realize the automatic parking of vehicles without human intervention, which is also an important step for the unmanned driving technology in practical applications. Vehicles or person in actual roads can be detected and classified with the aid of target detection technologies. Vehicles and person are also the main target objects to be detected on road by unmanned driving system using target detection technology.

As a specific application direction of target detection technology, vehicle target detection technology based on deep learning is not only used in unmanned driving system, but also has great application potential in intelligent transportation system. In recent years, with the increase of vehicle ownership in China year by year, the number of vehicles in China reached 281 million in 2020, with an increase of 21 million compared with that in 2019, presenting a year-on-year increase of 8.08%. By 2020, 70 cities had more than 1 million vehicles, 31 cities had more than 2 million vehicles, and 13 cities had more than 3 million vehicles. The huge number of preserved vehicles has brought a heavy burden to traffic roads; at the same time, it has also led to nearly 200,000 traffic accidents every year. An intelligent transportation system can be built by obtaining the corresponding information of road vehicles by using vehicle detection technology to identify vehicles, and then the whole transportation system can be controlled through communication, computer, and artificial intelligence technologies. The purpose of improving traffic efficiency and relieving traffic pressure can be achieved by extracting road information and intelligently dispatching vehicles.

With the improvement of people's material living standards, more and more people own private vehicles, which makes people have new and high demands for vehicles. Therefore, unmanned driving technology has become more and more concerned by people. The increase in the number of vehicles not only is convenient for people to travel, but also leads to some problems. Road congestion makes travel no longer convenient, and the demand for intelligent transportation has also attracted widespread attention. In recent years, the rise of deep learning and its wide application in the field of computer vision have stimulated the great progress of computer vision, and the computer vision technology has also been widely used in real life, such as automatic driving, face recognition, and image segmentation [1–3]. Both unmanned driving and intelligent transportation depend on vehicle detection. In this paper, the deep neural network is applied to vehicle detection, which is of great significance to automatic driving or intelligent transportation.

## 2. Related Works

As a kind of target detection technology, vehicle detection is identical to target detection in the main task objectives, which can be divided into target location and target classification. Vehicle detection algorithm has three main categories, including vehicle detection algorithm based on prior knowledge, vehicle detection algorithm based on shallow machine learning, and vehicle detection algorithm based on deep learning.

### 2.1. Traditional Vehicle Detection Algorithm

Like the traditional target detection technology, tradition-based vehicle detection algorithm needs manual design of target features. Among them, the detection algorithm based on prior knowledge identifies the vehicle through the lines, shadows, or some edge features of the vehicle body, and then extracts the position information of the vehicle in the image to achieve the purpose of vehicle detection through the difference between the gray levels of the shadow at the bottom of the vehicle and the surrounding pixels of the vehicle body. However, the effect of detection by this method will be greatly influenced by different lights, because the gray value of its image will be greatly influenced by light, and the shadow of nonvehicle objects similar to the shape and size of the vehicle will also be identical to that of the vehicle, so the algorithm will be misjudged, which is not suitable for high-precision detection. Vehicle detection by detecting vehicle brake lights is also achieved by artificially designing vehicle features. Vehicle detection can be realized by detecting vehicle brake lights, but its detection effect is not ideal enough because this method has great limitations due to the influence of light. The prior knowledge-based detection method uses the characteristics of the vehicle itself to carry out the detection task, but this kind of method has certain limitations and its detection recognition rate is not high, so it is difficult to meet the requirements of the detection task.

Traditional vehicle detection methods also include vehicle detection technology based on shallow machine learning, which realizes vehicle detection by combining machine learning algorithm on the basis of vehicle characteristics [4–6]. Detection accuracy can be improved by introducing SVM and HOG features by means of shallow machine learning, but this method also brings some problems while improving the accuracy. This method not only improves the detection accuracy through simple cascade, but also increases the scale of the model used for detection and the calculation amount accordingly. The addition of shallow machine learning method does improve the accuracy of vehicle detection to a certain extent, but this kind of method still relies on the selection of features. There is large amount of modeling work under complicated and changeable road conditions, which is the main reason that its development has been restricted. There are also some traditional vehicle detection algorithms such as frame difference method, streamer method, and background modeling method [7, 8]. This kind of algorithm can achieve certain recognition effect under specific conditions, but it also has many limitations, which are easily influenced by environmental factors, such as illumination and weather [9, 10]. Therefore, it is difficult to meet the real-time requirements of vehicle detection, and it is also unable to adapt to the increasingly complex road traffic environment.

### 2.2. Vehicle Detection Algorithm Based on Deep Learning

The vehicle detection algorithm based on deep learning is the same as the target detection algorithm based on deep learning, the methods employed are mainly classified into two categories, i.e., one-stage and single-stage target detection, and two-stage target detection can be available for judging whether there is recommended region or candidate region. One-stage target detection is wholly completed by one network through inputting images and outputting bounding box and classification label. Two-stage target detection is completed through two different networks through generating recommended regions by inputting images, and then sending them to a classifier for classification.

The representative algorithms of two-stage target detection include R–CNN, Fast R–CNN, and Faster R–CNN [11, 12]. The biggest feature of this method is that firstly, a certain number of candidate targets are generated based on regional recommendation, and then convolution neural network is used to process them. The R–CNN firstly conducts sparse sampling on the input original image by using candidate regions, then extracts features from the candidate regions by CNN, and finally classifies the extracted information by SVM (support vector machine). Compared with the traditional target detection algorithm, R–CNN has achieved significant improvement in the detection accuracy and the limitations of the algorithm have become much smaller [13, 14]. However, there are also many problems, among which the detection rate problem is rather obvious. This is because the network separately extracts features from a large number of candidate regions, which leads to a large number of repeated calculations conducted by the network, resulting in a lot of redundant calculation information and higher calculation cost. SPP-net adds a spatial pyramid pooling operation between convolution layer and full connection layer. In this operation, the features of the input images are extracted once to generate images with a fixed scale. However, the overall flow of the network still obtains candidate regions through region recommendation, then extracts Roi feature information of the images through CNN, and then carries out category judgment and position modification to achieve the purpose of detecting objects. However, because all the Roi feature information is obtained directly from the feature map, the operation of convolution is reduced to a large extent and the operation efficiency of the network is accordingly improved.

Through further optimization of SPP network, Fast R–CNN uses multi-task loss to replace the support vector machine (SVM) for classification, so that the regression of frame can also be trained through the network, and thereby classification and frame regression can be trained through the same network. However, the method of generating candidate region based on traditional methods needs to be processed on CPU, which limits the running speed of the system to a certain extent. Till the Faster R–CNN method was put forward, Faster R–CNN realized end-to-end target detection. The network extracts the candidate regions through RPN network and then shares the convolution layer with the generated candidate regions and the CNN which is classified. Firstly, multiple target candidate regions are generated by Faster R–CNN, then the features of target candidate regions are extracted based on region mapping and spatial pyramid pooling, and then various attributes of targets are identified in multiple branches led out by CNN in parallel. Compared with Fast R–CNN, Faster R–CNN accelerates the speed of region generation through the characteristics of RPN network [15, 16]. It classifies the detection target by judging whether the candidate box meets the feature requirements of the detection target first and then processing with the multi-task loss function.

The one-stage target detection algorithm is different from the two-stage detection algorithm. The one-stage target detection algorithm can directly calculate the classification and regression from multiple different positions of the image, so that the detection rate of the one-stage detection algorithm is better than that of the two-stage detection algorithm. YOLO series network, as the representative network of single-stage target detection algorithm, includes YOLO, YOLOv2, and YOLOv3 [17, 18]. These algorithms turn the target detection task into a regression problem by using the idea of regression, thus realizing the end-to-end identification of detection algorithms. YOLO network divides the input image into grids, in which each grid only needs to detect the target object whose center point falls on the grid, and then uses the anchor frame on each grid to replace the candidate frame in the two-stage detection network. This greatly improves the detection rate of the network and meets some tasks that require high real-time detection. By adding a network scale on the basis of the YOLOv3 series of end-to-end detection method to increase the connection between the convolution layer and the original convolution layer, the receptive field is expanded thereby, which makes the traditional YOLO series network have great advantages in identifying small objects. An SE-TinyYOLOv3 algorithm is an improved algorithm structure based on YOLOv3. This algorithm reduces the number of parameters of the model by redesigning the network structure of feature extraction of YOLOv3 algorithm, replacing the ordinary convolution layer with depth separation convolution layer, and then extracting richer feature information data from the trained sample data by broadening the lateral depth of the feature extraction network. The network can reduce the number of parameters without losing too much feature information, which makes the model have the characteristics of ensuring certain detection accuracy and real-time detection at the same time.

In the real road environment, the surrounding environment is complex and changeable, which requires high real-time performance of vehicle detection system. Target detection algorithm based on regional recommendation is the mainstream target detection algorithm at present, and its detection accuracy is also very high, which meets the requirements of vehicle detection system in accuracy. However, it has difficulty in meeting the requirements of roads with heavy traffic because of the large amount of calculation and the problem of detection rate of its model. For unmanned driving system, the speed of detection is more important. The target detection method based on regression is characterized by clear structure and good real-time detection. Although its detection accuracy is lower than that of the first method, it has better real-time performance for the vehicle detection system. Therefore, in practical application, one-stage detection algorithm is generally adopted as the vehicle detection algorithm. A neural network with 30 convolution layers is constructed by improving the basic network structure of DarkNet-53, which is a road vehicle target detection method based on YOLOv3 [19–21]. This network not only reduces the cost of training network, but also improves the detection rate of the network to a certain extent.

Real-time detection has always been an important research direction of vehicle identification, and an improved vehicle detection model based on the original YOLOv3 is also proposed for real-time detection of road vehicles. The improved network uses the inverse residual network as the basic feature extraction layer, so as to reduce the number of parameters, reduce the calculation amount and complexity of the model, and thus solve the problems of gradient disappearance and gradient explosion. At the same time, the improved network also uses group normalization to reduce the influence of batch data size on the accuracy of the model and reduces the number of missed detections by using the method of softening nonmaximum suppression, which not only ensures the real-time detection, but also takes into account the accuracy of detection. As for the problem of intelligent transportation, real-time problem of vehicle detection is also the focus of attention and research [22]. Some studies put forward a design basis with deep learning algorithm as the system and then design a vehicle tracking scheme with both real time and accuracy according to each actual scene, in which the real-time problem of vehicle detection serves as the key problem of the scheme design.

## 3. Design and Implementation of Vehicle Identification Based on YOLOv3

When detecting the vehicle target, there are the following problems for the vehicle dataset: small-sized target objects, the complexity of the vehicle environment, certain size scaling in the process of continuous detection, too many targets in a single image in the dataset, overlapping of targets, and other difficulties. In addition, vehicle detection has certain requirements for real-time performance of detection, so it is very important to choose a suitable detection algorithm. Although there are some difficulties, some common features of vehicles are obvious, for example, no matter what kind of vehicle, its wheels are basically round, and the most obvious feature of vehicles is the lines of the vehicle body. In this paper, a method based on deep learning will be adopted to realize vehicle detection.

### 3.1. Algorithm Selection Analysis

In practical application, the detection accuracy and speed of the target detection system serve as the key factors to be considered when designing the algorithm. The higher the detection accuracy, the stronger the ability to detect objects will be; the faster the detection rate, the greater the practicability of applying it to practical products.  Table 1 shows the concrete performance of several common target detection algorithms in detection rate and detection accuracy.

From Table 1, we can see that Faster R–CNN has a good performance in detection accuracy, but the detection rate is quite different from that of several one-stage detection networks. These one-stage detection networks do not have bad performance in the detection rate, and it is obviously better than the detection algorithm Faster R–CNN in the second stage. As for the accuracy of detection, YOLO is slightly inferior. Considering the problems mentioned above, YOLOv3 is better in detecting small-sized objects, and it has a good performance in detection accuracy and detection rate, so YOLOv3 is chosen as the vehicle detection algorithm in this paper.

### 3.2. Model Design

#### 3.2.1. Initialization Operation of Candidate Box

Training the network is the key to the whole detection task, and some parameters need to be initialized before training the network model. The initialization of candidate box size is one of the most important initialization operations. The quality of candidate box initialization will affect the training time and training effect, because the training and testing of the network need to be carried out on the basis of initial candidate box initialization. In YOLOv3, the size of the candidate box is initialized by using *k*-means. The evaluation index of *k*-means clustering algorithm is the value obtained on the basis of Euclidean distance. The so-called Euclidean distance index means that for two targets, the smaller the Euclidean distance between them, the higher the similarity between the two targets will be and vice versa. For *k*-means clustering algorithm, at first, it is necessary to determine several points as the center points of clustering and then calculate the value of Euclidean distance from other points or other targets to these clustering centers. The one with the smallest Euclidean distance between the target and the clustering point is the category to which the target belongs, and then it is required to move the clustering center point to the center position of the category. At this point, the operation is completed once, and then such iteration is repeated for a certain number of times until the center point no longer moves, so as to achieve the clustering of targets.

For YOLOv3, the idea of employing k-means is for clustering the bounding box. For each image used for training, there are several marked bounding boxes. The first step in bounding box clustering is to take out all bounding boxes in the images used in training and put them together. As the clustering of bounding box needs to use the elements of width and height of the box, but for the original data, width and height are contained in the coordinates of two points of the box, that is, the coordinates of the upper left corner and the lower right corner, it is necessary to obtain the *W* and *H* values of the box through these two coordinate values. After processing, it is required to select *K* values in all bounding boxes as the clustering values of anchor box clusters, that is, the initial values of boxes, and *K* is selected as 9 in this paper.

#### 3.2.2. Detection Module of Network

The backbone network used by YOLOv3 is DarkNet-53, through which the features of the input data can be extracted. The deep-level network structure is beneficial to the network extracting more feature information, but there are also some problems for the network that resides in too deep level. Deep-level network will lead to the lack of feature information of small-sized objects, which will result in the decline of the network detection ability for small-sized objects, which is also the problem of several other one-stage detection networks. However, based on the idea of residual network, DarkNet-53 further improves the learning ability to image features by using residual connection, and at the same time, it also makes up for the shortcomings in the detection on small-sized objects.

The design of loss function plays a very important role for each detection network. The design of a loss function will determine the training result of the model.

In case of the maximum IOU value between the predicted frame and the real frame generated during training, the target shall be marked as a positive sample and included in the loss function. For the anchor frame without the maximum IOU value, the target shall not be included in the loss function. Therefore, for each existing real frame, there is only one generated prediction frame that corresponds to the real frame one by one. The whole loss calculation includes loss of confidence, loss of category, and loss of anchor frame coordinates.

The loss of confidence is mainly expressed as whether a certain cell in the detection layer contains the target center point, namely, the target object.

## 4. Experiment Results and Analysis

### 4.1. Selection of Dataset

The selection of dataset is the most critical step in designing a target detection system by using deep learning method. In this paper, we select the image dataset in BDD100K, as the input data for model training.  Figure 1 shows some part of data in the dataset.

The data images contained in this dataset are all road vehicles photographed by driving vehicles, including different types and numbers of vehicles and person, and other targets. The whole dataset contains a total of ten categories of target objects, and we only used six categories in the dataset, specifically cars, buses, pedestrian, trucks, motor, and bikes.

### 4.2. Data Processing

The downloaded data are classified into image part and label part. For the newly downloaded data stored in JSON format as indicated on label part, each JSON file corresponds to an image with the same file name. This file contains the name of the corresponding image file, as well as the category information, category name, and position information of the marked box in the image. The location information includes two points, that is, the horizontal and vertical coordinates of the top left corner of the box and the horizontal and vertical coordinates of the bottom right corner of the box, through which the position of the box can be determined. At the same time, one image can contain multiple boxes.

It is difficult to directly use the contents in JSON format file, which contains some redundant information. Thus, it is necessary to transform the file in this format to simplify the information structure and eliminate redundant information data at the same time. First, it is required to convert JSON-formatted files into xml-formatted files. Compared with the original JSON file, the processed file is much simpler in structure and contains more concise data information. At the same time, the width and height of the image and the location of the file are properly written into the file.

The processed xml file cannot be directly used as input data for training, and such processed xml is actually equivalent to the file generated after tagging by tagging software. However, the input data for training need simpler format input, and redundant descriptions in the file need to be further removed. Finally, only the path of the image file, the position of the box in the image, and the category of the object in the box are retained. At last, the data need to be processed into a text file with txt suffix as its format, using the absolute path of the image and the corresponding image name, and containing the position of the box contained in the image and the category information of the box. The processed txt file contains the data information of all the images used in training. The images that need to be input can be found through the absolute path, which is followed by the contents of the inner box of the images. Thereby, all the required images and data can be integrated through a. txt file to facilitate the network to read the data.

### 4.3. Model Detection

Model training is the last step to realize the vehicle detection model, and the final detection task can be carried out by loading the trained weight on the model. Some parameter settings of the training process are as shown in Table 2.

In the task of training or detection, YOLOv3 is mainly used for target detection of three characteristic layers in the backbone network, which are located in the bottom layer, middle lower layer, and middle layer of the backbone network.

### 4.4. Results and Analysis

Training the detection network needs to set some parameters to ensure that the trained model can have good performance. In the YOLOv3 detection algorithm used in this paper, the learning rate setting actually has two values of 1 *e* − 3 and l *e* – 4, respectively. The learning rate is changed by the method of breakpoint continuation, i.e., first training the model by large learning rate and then optimizing the model by using small learning rate. The epoch value is set to 50. Of course, if the model can continue to be optimized, the method of breakpoint continuation can also be used to retrain the epoch for a certain number of times. The value of loss after training is shown in Figure 2.

The blue curve in the figure represents the loss value of the training set, and the orange curve represents the loss value of the test set. The loss values at the beginning of training are particularly large, the loss values in several epochs at the beginning of training drop very sharply, and then the falling speed slows down and then tends to converging. Although the loss value after training is still relatively large intuitively, the comparison shows that the model has been converging. The loss value of the training set basically presents stable decreasing and tends to be stable at last and then oscillates within a certain range. It is required to continue training by changing the learning rate with the method of breakpoint continuation, but the performance of training results is not much different from those of the second half of Figure 3.

Map value is an important index to measure a target detection model. Each category has an ap value to be used as the recognition effect of the detection network for that category, while map is the average of all categories of ap. The map value of the model trained in this paper is 72.8. Numerically speaking, its performance is slightly lower. As far as the detection effect is concerned, the detection effect of cars is still very good, but the detection performance of buses and motors is relatively poorer.

From the results shown in Figure 3, it can be seen that most of the detection of the car category by the model is good, and the scores of the detection boxes are mostly kept above 0.7. The detection effect of trucks is not too bad, but the detection effect of bus categories is a little worse, and the score of detection box is mostly not high.  Figure 4 shows the detection effect of the network on bike category and person category.

From the results in Figure 4, it can be seen that the detection effect of the detection model on bike category and person category is also not bad, but relatively speaking, the score for person category is higher and that for bike category is relatively lower. And the detection box for person category is more accurate and the box selection is more comprehensive.

From the detection results in Figure 5, the detection effect of bus category is general. Although it can be detected as bus category, there are only three buses identified in the figure on the left, and only the first bus has a higher score. On the other hand, it can be seen from the right figure that the box of bus category is not particularly complete, resulting in part of the vehicle body being out of the detection box.

As far as the detection effect is concerned, the detection effect of person category is much better, and the detection effect of motor category is slightly worse. In terms of scores, other score on person category is also significantly higher.

The detection accuracy of the model used in this paper is relatively good in terms of the overall detection, especially the car category and person category, which have the best detection effect, but the detection accuracy for motor category and bus category is acceptable, and the detection box is slightly insufficient. Reasons: There are millions of targets in the car category, but there are only over 10,000 targets for bus category, and the motor category has even less targets, only over 4,000. As a result, most of the data trained by the model during training are of car category, most of the features extracted are the feature information of car category, and most of the parameters modified during reverse feedback tend to be modified in a direction that is beneficial to the detection on car category. This is also why the accuracy of the detection on the car category remains relatively high. For the person category, the number of targets has reached 100,000; that is, it has a high proportion in training. At the same time, the feature information of the person category is quite different from that of various vehicles, which also makes the detection effect of the person category much better.

## 5. Conclusions and Future Work

With the development of artificial intelligence technology, more and more industries will use technologies of AI. The artificial intelligence technology based on deep learning has also made great progress thereby. The excellent performance of deep learning technology in image aspect makes a breakthrough in target detection. In recent years, the popularization of unmanned driving vehicles and the proposal of intelligent transportation have caused extensive research on vehicle target detection.

For traditional vehicle recognition, neither the performance nor the efficiency of detection can adapt to the rapid development of unmanned driving technology or the application of intelligent transportation. Vehicle detection based on deep learning can detect vehicle targets by means of deep learning, which can better adapt to the current rapidly developing technology and complete the detection task more effectively.

In this paper, the vehicle target detection based on deep learning is studied. Although the final detection effect is not bad, there is still room for further improvement. First of all, the use of data is not well balanced. Although the detection effect of a certain category is good, it causes the network to pay more attention to the characteristics of this category, which reduces the detection effect of other categories. Furthermore, more kinds of algorithms shall be made available for use in detection, and the vehicle detection model obtained by deep learning can be comprehensively analyzed by multiple algorithms.

## Figures and Tables

**Figure 1:** BDD100K data image.

**Figure 2:** Loss value of YOLO training.

**Figure 3:** Diagram of the detection on road vehicles.

**Figure 4:** Diagram of the detection on bike category and person category.

**Figure 5:** Detection effect on bus category.

**Table 1:** Evaluation diagram of common detection algorithms.

Algorithm	Training set	Test set	MAP	fps
Faster R–CNN	VOC2007 + 2012[19]	2007	73.2	17
YOLO	VOC2007 + 2012	2007	63.4	45
SSD	VOC2007 + 2012	2007	74.3	46
YOLOv3	VOC2007 + 2012	2007	76.1	50

**Table 2:** Parameter settings.

num_classes	6
Lr	1 *e* − 3
batch_size	32
Input_ship	(416,416)

## Data Availability

The data used to support the findings of this study are available from the corresponding author upon request.
